The article "Examining the Relationship Between Product Market Competition and Chinese Firms Performance: The Mediating Impact of Capital Structure and Moderating Influence of Firm Size" was retracted in 2025. Reasons: unreliable results or conclusions; a conflict of interest; concerns about the peer review; concerns about the citations.

# Examining the Relationship Between Product Market Competition and Chinese Firms Performance: The Mediating Impact of Capital Structure and Moderating Influence of Firm Size

**DOI:** 10.3389/fpsyg.2021.709678

**Published:** 2022-05-17

**Authors:** Riaqa Mubeen, Dongping Han, Jaffar Abbas, Saqlain Raza, Wang Bodian

**Affiliations:** ^1^School of Management, Harbin Institute of Technology, Harbin, China; ^2^Antai College of Economics and Management, Shanghai Jiao Tong University, Shanghai, China; ^3^School of Media and Communication, Shanghai Jiao Tong University, Shanghai, China; ^4^Faculty of Management Sciences, Shaheed Zulfikar Ali Bhutto Institute of Science and Technology, Islamabad, Pakistan; ^5^School of Economics and Management, Harbin Institute of Technology, Harbin, China

**Keywords:** product market competition, GMM model, firm size, capital structure, firm performance

## Abstract

This study emphasized the relationship between the Chinese companies’ product market competition and organizational performance. This article explored the mediating effect of capital structure and the moderating impact of firm size in achieving better performance of Chinese companies. This study employed a sample of 2,502 Chinese firm observations and identified that market competition positively influenced firm performance. Additionally, capital structure partly mediated the relationship between product market competition and firm performance. Similarly, the present study also tested the moderating effect of firm size (both small and large) on the association between product market competition and firm performance. The results showed that moderating large businesses affects the nexus between product market competition and firm performance. Conversely, small firms’ moderating role revealed a substantial adverse impact on the association between product market competition and firm performance. These findings contribute to the literature on the complex implications of market competition on business firms’ performance. The results provide insightful and practical implications for future research directions.

## Introduction

Many organizations consider corporate competitive strategies to be a strategic imperative in an increasingly competitive global environment. Corporate competitive strategies are those corporate plans firms use to increase market share (Franko, 1989), competitive advantage (Hitt et al., 1996), and improve firm performance (Giroud and Mueller, 2011). Businesses incorporate competitive strategies as an essential tool to achieve their objectives. Many scholars have long been interested in investigating corporate strategy, and they focused on examining the relationship between product market competition and firm performance (Raith, 2003; Pant and Pattanayak, 2010; Sheikh, 2018; Javeed et al., 2020). Existing studies revealed mixed findings on this relationship. Previous studies (Raith, 2003; Pant and Pattanayak, 2010; Sheikh, 2018) reported that competition positively and significantly affects firm performance (Mubeen et al., 2020). However, another study showed that business competition forms a competitive setting for businesses, decreasing pricing power and thus leading to low profits (Javeed et al., 2020). The consequences of the impact differ significantly due to the different data, time, and various performance measurements. Consequently, academics recommend that the intervening mechanism between product market competition and firm performance be studied to uncover whether and how product market competition affects firm performance (Sheikh, 2018). However, few studies have examined the intermediate link between product market competition and company performance, leading the authors to suggest that intervention variables should be explored in future studies. Another study (Michaelides et al., 2019) debated that the impact of competition may be limited or enhanced depending on the organizational environment. In reality, several aspects of the corporate business environment may moderate or mediate the relationship between product market competition and firm performance, such as organizational capital structure, firm size, growth orientation, and ask requirement (Blundell et al., 1999; Guney et al., 2011; Ammann et al., 2013; Dang et al., 2018). For example, researchers have called for more research on the contingencies—moderators and mediating mechanism affecting the product market competition and firm performance relationship. Therefore, we explore this question by examining how product market competition affects firm performance through the two mediating and moderating mechanisms: capital structure and firm size.

The article "Examining the Relationship Between Product Market Competition and Chinese Firms Performance: The Mediating Impact of Capital Structure and Moderating Influence of Firm Size" was retracted in 2025. Reasons: unreliable results or conclusions; a conflict of interest; concerns about the peer review; concerns about the citations.

We focus on capital structure and firm size as intervening mechanisms in this study because prior literature indicates that these two variables are significant predictors of organizational values (Hillman et al., 2007; Gul et al., 2011). Research has theorized and empirically found that capital structure is a valuable resource that enables a business to generate higher firm value. Additionally, scholars considered firm size a critical underlying mechanism between product market competition and firm performance, constraining or facilitating business activities such as decision making and firm innovation process (Li and Chen, 2018).

Capital structure works as a valuable source for earning higher profits by producing high-quality or value products for the competitive markets (Boubaker et al., 2018). This study examines the direct impact of market competition on capital structure and investigates the mediating role of capital structure on the association of market competition to attain firm performance. Existing literature debated that capital structure cannot be neglected in a competitive organizational environment (Jiraporn et al., 2012). According to the authors’ knowledge, no study is available that investigates the mediating impact of capital structure on the association of market competition and firm performance. Therefore, this is the first study highlighting the role of capital structure on the relationship between market competition and firm performance. However, the present study emphasizes the moderating effect of firm size based on the following arguments. First, firm size is important for organizational performance and management. Managerial productivity increase with firm size (Zona et al., 2013; Dang et al., 2018). For example, larger firms are more advanced and well-organized to respond to market changes for achieving the desired profit.

This study focused on examining product market competition and firm performance in the Chinese economy. Next, it investigated capital structure as a mediating factor in this relationship. Furthermore, it used the firm as a moderating factor to study the connection between product market competition and firm performance. Using the GMM model, the results revealed that the product market competition positively connects with firm performance, and capital structure partially mediates this relationship. Furthermore, small firms negatively affect this relationship, while large firms positively moderate the connection between product market competition and firm performance. Therefore, it is essential to consider this variable to evaluate the relationship between market competition and firm performance.

In brief, this study offers two significant contributions to the association between market competition and firm performance. First, we test whether capital structure mediates the market competition and firm performance association. Second, this study tests the moderating role of firm size on this relationship because, before this, most studies investigated only product market competition and firm performance (Yuan et al., 2019). This study promotes the role of market competition in China and other developing economies.

The research classification specifies the subsequent sections. Section “Literature Review” introduces the literature, theoretical framework, and hypothesis development. Section “Research Data, Sample, and Methods” provides detailed information on sample and variable selection. It describes applicable econometric techniques. Section “Results and Discussion” provides the results of this research and discussion. Finally, Section “Discussion” summarizes the research and policy implications. Figure 1 displays the conceptual framework of the study.

The article "Examining the Relationship Between Product Market Competition and Chinese Firms Performance: The Mediating Impact of Capital Structure and Moderating Influence of Firm Size" was retracted in 2025. Reasons: unreliable results or conclusions; a conflict of interest; concerns about the peer review; concerns about the citations.

**FIGURE 1:** Conceptual framework of the study.

## Literature Review

### The Relationship Between Product Market Competition and Firm Performance

Several theoretical literature debated that strong product market competition leads to better understanding and improved performance. As market competition builds a better reputation, it provides competitive benefits, and these advantages are consequences of increased firm values. As the main goal of an enterprise is to achieve higher financial returns, attaining a sustainable competitive advantage plays a vital role (Dunk, 2007). Accordingly, many corporate strategies aim to gain a sustainable competitive advantage. The competitive scenario builds an excellent image for businesses in a competitive market and provides competitive advantages (Saeidi et al., 2015). Competitive advantage enables the firm to gain higher firm value by offering superior products and services.

Additionally, the literature indicated that product market competition is a powerful force that solves agency conflicts between owners and managers and reduces the managerial slack, leading to increased firm values (Hermalin, 1992; Mnasri and Ellouze, 2015; Li M. et al., 2018; Abbas et al., 2019b; Javeed et al., 2020). Managers in competitive industries face more bankruptcy risk than those in concentrated industries do. Therefore, managers are prompted to make the best and worthy decisions due to the fear of losing their jobs (Abbas et al., 2020; Aman et al., 2021b; Fu and Abbas, 2021). Another study contended that pressure is essential for enhancing firm performance (Ammann et al., 2013). Empirical studies showed the positive and negative association between product market competition and firm performance. For instance Ammann et al. (2013) explained that competition works as the desired tool for shareholders because it influences top management to work hard. Therefore, it reduces agency costs, increasing profitability.

For instance, a study of 670 United Kingdom companies from 1972 to 1986 showed that competition was positively correlated with organizational performance. Additionally, various researchers have studied the relationship between corporate performance and competition. A previous study (Januszewski et al., 2002) examined the association between product market competition, corporate governance in Germany by selecting 500 firms from 1986 to 1994. Their findings showed that product market competition positively affects productivity and strong competition compels businesses to convert resources into social profit maximization (Fernández-Kranz and Santaló, 2010). Moreover, previous research evidence that competition is positively related to firm performance (Okada, 2005), while other studies identify a non-linear link between competition and firm values (Tingvall and Poldahl, 2006; Inui et al., 2012). Consequently, some previous works concluded that there is an inverted U-shaped association between competition and firm profit.

The article "Examining the Relationship Between Product Market Competition and Chinese Firms Performance: The Mediating Impact of Capital Structure and Moderating Influence of Firm Size" was retracted in 2025. Reasons: unreliable results or conclusions; a conflict of interest; concerns about the peer review; concerns about the citations.

When referring to some literature examined in emerging economies, we noticed that their results are conducive to the positive connection between product market competition and performance. For example, Javeed et al. (2020) investigated the association between product market competition and firm performance and selected 147 Pakistani firms’ data over 2008–2017. Their findings showed that product market competition has positive effects on company performance. Other studies have tested the link between product market competition and firm value, and the results revealed the positive connection between product market competition and firm value concentration (Blundell et al., 1999). Sattar et al. (2020) also reported a positive relationship between firm value and product competition. Based on the literature review, we established the Hypothesis as follows:

**H1**: Product market competition has a positive effect on firm performance.

### The Relationship Between Product Market Competition and Firm Performance With Mediating Effects of Capital Structure

Numerous experimental studies have revealed that the effect of firm market competition on firm performance may change based on the strength of the corporate debt structure. These studies conclude that market competition has a complex interaction with the firm’s debt structure. For instance, Brander and Lewis (1986) recommend that capital structure or debt allows organizations to compete in highly competitive environments. Furthermore, it is always a top priority for managers to increase the leverage, reducing agency problems between managers and shareholders, and leading to higher profits. Thus, capital structure is vital for business growth and to achieve the defined firm strategic objectives.

Capital structure and company performance have attracted much empirical debate, and the results of empirical studies are mixed. For example, advocates of agency theory believe that a company’s capital structure negatively impacts financial performance (Margaritis and Psillaki, 2010; Chintrakarn et al., 2014). However, limited liability and disciplining effect proposed a positive impact of leverage on performance (Brander and Lewis, 1986; Fosu, 2013). Capital structure is considered outside funding that permits a firm to advance more products, thus positively impacting firm performance (Jiraporn et al., 2012). In contrast, leverage will enable organizations to participate more aggressively in the market due to limited liability. A previous study debated that different conditions impact the profit of such planned behavior on the type of competition and product features (Wanzenried, 2003). It recommends that leverage effects could fail to increase leveraged business effectiveness. Previous literature suggests that leveraged firms could suffer significant competitive disadvantage in product markets (Chevalier, 1995; Wanzenried, 2003).

The article "Examining the Relationship Between Product Market Competition and Chinese Firms Performance: The Mediating Impact of Capital Structure and Moderating Influence of Firm Size" was retracted in 2025. Reasons: unreliable results or conclusions; a conflict of interest; concerns about the peer review; concerns about the citations.

Capital structure is an organizational plan that enables a company to gain a competitive benefit by adding other products to increase company performance (Desai et al., 2003). Therefore, we hypothesize that Capital structure is an essential mediating variable in understanding how market competition is related to firm performance. This is because the intermediary variable plays a vital role in organizational sciences. It is useful to examine the association between product market competition and firm performance by adding mediation and intermediator, and how and why one variable impacts another (Franko, 1989). Existing literature has empirically found that managers prefer high leverage, which raises profits and positively impacts firm performance (Fosberg, 2004). Other studies have also found that market competition is positively related to durable firm performance (Abor, 2007). Furthermore, existing literature demonstrates that leverage opens up opportunities for rivalry predation in concentrated product markets, increasing firm growth and profits (Chevalier, 1995; Dasgupta and Titman, 1998; Fosu, 2013). Based on the above-stated literature review, we propose the following hypothesis:

**H2**: Capital structure mediates the relationship between product market competition and firm performance.

**H2a**: Product market competition is negatively associated with capital structure.

**H2b**: Capital structure positively mediates the relationship between market competition and firm performance.

### The Relationship Between Product Market Competition and Firm Performance With Moderating Effects of Firm Size

The literature demonstrates that the association between product market competition and firm performance has produced mixed outcomes (Fosu, 2013; Sheikh, 2018; Javeed et al., 2020). However, minimal evidence shows why these results are so different in the literature. Sheikh (2018) explained that some organizational factors might not allow the firm to achieve the benefits of market competition. The literature recognized firm size as one of the moderating mechanisms, which may modify business activities to fulfill their objectives, such as managers’ interests, firm improvement, and decision making (Januszewski et al., 2002; Li and Chen, 2018). This study investigates whether firm size plays a moderating role in improving or constraining the effect of product market competition and firm performance. However, no empirical research found how and why firm size might enhance or restrain the association of product market competition and firm performance. Therefore, we employ firm size as a moderating element to explain why observed conclusions on the product market competition and firm performance are seemingly contradictory.

The article "Examining the Relationship Between Product Market Competition and Chinese Firms Performance: The Mediating Impact of Capital Structure and Moderating Influence of Firm Size" was retracted in 2025. Reasons: unreliable results or conclusions; a conflict of interest; concerns about the peer review; concerns about the citations.

Existing literature on market competition demonstrates that large firms have strong market reputations and more assets to produce new products. Although theoretical recommendations were made that market competition may change over firm size (Dang et al., 2018), these suggestions lead to possible pressure between firm size and market competition as they are linked with firm performance (McWilliams et al., 2006). For instance, larger firms have more resources and market reputation than smaller firms do. Additionally, they are more skilled in producing new products and achieving desired goals (Damanpour, 2010; Zona et al., 2013).

In general, larger firms are more advanced and well-organized to respond to market changes (Rajan and Zingales, 1995). However, smaller firms have low resources, and their organizational structure is not well-organized. Additionally, smaller firms with insufficient resources cannot produce according to market changes. They tend to utilize accessible resources to increase their performance (Baker and Hall, 2004). Based on this discussion, we hypothesize that firm size is an important variable to understand how market competition increases firm performance (Yang and Zhao, 2014). Furthermore, it discloses how and why one variable affects another (Baron and Kenny, 1986). Thus, we establish the following hypothesis:

**H3**: Firm size moderates the association between product market competition and firm performance.

**H3 (a)**: There is a positive relationship between product market competition and firm performance when firm size is large.

**H3 (b)**: There is a negative association between product market competition and firm performance when firm size is small.

## Research Data, Sample, and Methods

We collected data from the Chinese stock market and accounting research (CSMAR) database and spans 2012–2017 due to lack of data and missing values. The study considered a panel dataset from Chinese listed firms over 2012–2017. The reason behind the data period (2012–2017) are as follows, For instance, the china securities regulatory commission (CSRC) 2006 has focused on the improvement of organizational structure as a priority (Li and Chen, 2018). In response to deepening market development, Chinese firms have gradually implementing corporate governance structures, especially many measures adopted (Conyon and He, 2011). Second, we excluded the financial crises duration (2008–2009) as mentioned (Kirkpatrick, 2009; Kahle and Stulz, 2013). For the study analysis we focused on state-owned enterprise firms as we collected data from CSMAR database which includes only publicly listed firms rather than all Chinese firms (Liu et al., 2018). This study contains a sample of manufacturing firms’ annual observations, and the data filtering techniques have been employed; therefore, it ignores organizations with incomplete data. Additionally, we select firms with at least 3 consecutive years’ statistics for the GMM regression analysis. Finally, we used 417 firms covering 6-year data, with 2,502 firms’ years’ observations. We chose the Chinese economy because it has achieved immense success amongst emerging countries and has done detailed work on the role of corporate governance.

The article "Examining the Relationship Between Product Market Competition and Chinese Firms Performance: The Mediating Impact of Capital Structure and Moderating Influence of Firm Size" was retracted in 2025. Reasons: unreliable results or conclusions; a conflict of interest; concerns about the peer review; concerns about the citations.

The reason behind the data period (2012–2017) are as follows, For instance, the china securities regulatory commission (CSRC) 2006 has focused on the improvement of organizational structure as a priority (Li and Chen, 2018). In response to deepening market development, Chinese firms have gradually implementing corporate governance structures, especially many measures adopted (Conyon and He, 2011). Second, we excluded the financial crises duration (2008–2009) as mentioned (Kirkpatrick, 2009; Kahle and Stulz, 2013). For the study analysis we focused on state-owned enterprise firms as we collected data from CSMAR database which includes only publicly listed firms rather than all Chinese firms (Liu et al., 2018).

### Variable Definition

#### Product Market Competition

Product market competition is the main independent variable in our study. In terms of operations, the degree of product market competition means the monopoly, oligopoly, or competitiveness of the company. Existing studies have used different techniques to measure market competition, such as the Herfindahl Hirschman Index (HHI) and Boone Index (Fosu, 2013). Previous research has shown that HHI is the best measure of market competition among other available methods (Zou et al., 2015). Past research has also shown that companies usually compete based on their sales, indicating the industry’s competition in terms of revenue (Zou et al., 2015). Additionally, many scholars have used the HHI to calculate industry competition (Jain et al., 2013; Michaelides et al., 2019). Following (Michaelides et al., 2019; Javeed et al., 2020), we use each company’s total squared market share in the industry to calculate market competition based on the total sales of the industry.

The article "Examining the Relationship Between Product Market Competition and Chinese Firms Performance: The Mediating Impact of Capital Structure and Moderating Influence of Firm Size" was retracted in 2025. Reasons: unreliable results or conclusions; a conflict of interest; concerns about the peer review; concerns about the citations.

#### Firm Performance

In this study, we use company performance as our dependent variable. Existing literature showed that various methods could be used to calculate company performance, such as return on assets (ROA), return on investment (ROI), return on equity (ROE), Tobin Q, and dividends payable (Javeed et al., 2020). However, we use ROA and ROE measures as our dependent variables. Some studies (Hutchinson and Gul, 2004; Javeed et al., 2020) reported that accounting-based measurement methods are most suitable for corporate governance research because they can easily track the company’s ability to manage its value. By adding to this debate, Bhagat and Bolton (2008) indicated that a higher ROA reflects the organization’s aptitude on asset efficiency and shareholder value.

Furthermore, ROA discloses firm production related to management when using assets. Therefore, based on previous research, we calculated the ROA by the ratio of the firm’s net profit to total assets (Javeed et al., 2020). While the calculation method of ROE is the ratio of operating profit to shareholder’s equity (Bhagat and Bolton, 2008), ROE is mainly used for corporate governance-related research and research related to corporate governance. According to the shareholders’ perspective, return on equity has better tested the company’s business performance (Brown and Caylor, 2009).

#### Control Variables

This study used different control variables to obtain more relevant results: growth, current ratio, and innovation. Companies with high growth expectations will have realistic opportunities for future profits and flexibility in choosing future investments, so the rate of return may be positively correlated with growth. Sales growth (Growth), a proxy for growth opportunities, was measured as changes in the company’s sales revenue (King and Santor, 2008). The current nature of assets (liquidity) can improve the company’s solvency; therefore, the relationship between debt and current ratios can be positive or negative. The current ratio is calculated by dividing total existing assets by total current liabilities (Guney et al., 2011). We use R&D expenses (research and development expenses) for the innovation measurements as a proxy for innovation. Scholars believe that innovation reflects management decisions; allocating resources to produce more products, and previous literature has proven that the company’s R&D intensity is an appropriate proxy for the firm’s innovation (O’Brien, 2003; Miller and Del Carmen Triana, 2009). Consistent with this, innovation is measured by the intensity of R&D. We use this as the company’s reported R&D expenditure divided by sales (Miller and Del Carmen Triana, 2009).

The article "Examining the Relationship Between Product Market Competition and Chinese Firms Performance: The Mediating Impact of Capital Structure and Moderating Influence of Firm Size" was retracted in 2025. Reasons: unreliable results or conclusions; a conflict of interest; concerns about the peer review; concerns about the citations.

#### Moderating and Mediating Variables

Existing literature indicates intervening variables in the relationship between gender diversity and firm performance (Fosu, 2013). To address the concerns, we investigated the moderating and mediating role of firm size and capital structure on the association between product market competition and firm performance. This study used the capital structure as a mediating variable to investigate their mediating role in the association between product market competition and firm performance. For the mediation analysis, the capital structure may be defined in various ways. Previous work debates that the definition of the capital structure depends on the study objective (Rajan and Zingales, 1995). In this study, we define capital structure as the ratio of total debt to total assets.

In the corporate finance literature, firm size is a crucial variable. Existing studies used firm size as a control variable in all studies of corporate finance. However, this study used moderating variables based on the identified current literature gaps that firm size should be studied in the association between product market competition and firm performance. Firm performance is not the same at different firm sizes. Previous work demonstrates other methods to measure firm size, such as total sales, natural log of total assets, and market equity assets (Dang et al., 2018). Following a current study, we used firm size as a log of total sales (Dang et al., 2018).

### Empirical Examination

In the regression model, when there is a correlation between the error terms, the variables face endogeneity problems. Similarly, these problems may also result from automatic regression or missing variables, measurement errors, and autocorrelation errors (Singh et al., 2018). According to the rules of econometrics, if there is only one endogenous variable in the research model, appropriate techniques need to be applied to solve the endogenous problem (Javeed et al., 2020). Endogeneity correlates explanatory variables with error terms (Cannella et al., 2008). The formation of the panel dataset places limitations using OLS (ordinary least square model) because it leads to biased estimation and unobserved heterogeneity (Javeed et al., 2020). For example, dealing with historical company information, such as unobservable and observable company characteristics, leads to endogenous issues (Kang and Zardkoohi, 2005). Unnoticeable heterogeneity, dynamic, and simultaneity endogeneity are multiple causes of endogeneity. According to scholars, about 90% of the research published in reputable journals has not yet fully discussed the issue of endogeneity (Hamilton and Nickerson, 2003; Antonakis et al., 2010; Javeed et al., 2020). Therefore, literature suggested that it needs to tackle endogenous problems.

The article "Examining the Relationship Between Product Market Competition and Chinese Firms Performance: The Mediating Impact of Capital Structure and Moderating Influence of Firm Size" was retracted in 2025. Reasons: unreliable results or conclusions; a conflict of interest; concerns about the peer review; concerns about the citations.

Existing studies argued that there are many techniques to solve the endogenous problems in panel data. The literature reported that control variables could solve the three-factor effect (Li, 2016). Additionally, the lagged independent variable is a crucial method to overcome the simultaneous issues. Nevertheless, to eliminate causality, tool change technology is considered a top priority. Moreover, lagged dependent variable techniques can deal with solid historical information such as unobservable and observable effects. After studying all approaches to deal with the endogeneity issue, like using variables to control the firm fixed effects, third-factor effects, lagged independent variables, and GMM or dynamic models controls upward. Downward bias, and in certain situations in OLS assessment (Li, 2016), most scholars propose the generalized method of moments (GMM). The GMM model is a superior technique to overcome endogenous problems (Wintoki et al., 2012). In this study, we used GMM model heteroscedasticity and autocorrelation, and endogeneity issues.

Arellano and Bond (1991) first proposed the GMM, explicitly used for panel data (Arellano and Bond, 1991). For dynamic panel data, the causality of primary sight usually changes over time. In this case, this technique is suitable for the lag of the predictor variable as an independent variable. Therefore, the lag value of the predictor variable is considered as a tool to overcome endogeneity. Furthermore, the GMM model overcomes endogeneity by “inner altering the data” -when a variable’s initial value is subtracted from the current value, the change implies a statistical situation (Wooldridge, 2016). Finally, GMM is a suitable approach for controlling endogenous problems than other methods. GMM has a higher effect on coefficient correction (Javeed et al., 2021).

We used some specific tests to check whether data is appropriate for examination before applying the GMM model. First, this study used a variance inflation factor (VIF) test to confirm the multicollinearity issues in data. The results of the VIF test guaranteed that there are no multicollinearity issues in this study. Next, this study applied the Wald test to check for heteroscedasticity. The outcomes of the Wald test display no heteroscedasticity in this data. The study used the Sargan test for instrument validity and over-identifying restrictions. Sargan test outcomes confirm the validity of instrumental variables. This study established the data for serial autocorrelation by applying an AR (1) and AR (2) test and concluded no serial autocorrelation. Finally, we tested the data for endogeneity problems and found that our data have endogeneity issues. This study incorporated the GMM model to explore endogeneity problems between variables and error terms. The study examined the consistency of the GMM model with previous research, which stated that GMM is the best model among other statistical analytical techniques (Singh et al., 2018). Hence, the GMM model is a superior method with the maximum power to deal with endogeneity (Javeed et al., 2020). All instrument tests show that the weak instruments do not affect the study’s specifications, and instrumental variables perform well.

The article "Examining the Relationship Between Product Market Competition and Chinese Firms Performance: The Mediating Impact of Capital Structure and Moderating Influence of Firm Size" was retracted in 2025. Reasons: unreliable results or conclusions; a conflict of interest; concerns about the peer review; concerns about the citations.

## Results and Discussion

### Descriptive Statistics

Table 1 describes the descriptive statistics and VIF of all dependent and independent variables of this study (Abbas et al., 2019a,c). Panel A shows the descriptive statistics of the data, and this study applied ROA and ROE as dependent variables based on the total 2,502 observations used in 5 years (Hussain et al., 2019, 2021). All details of descriptive statistics of all variables are given in panel A.

**TABLE 1:** Analysis of variance inflation factor (VIF).

	Panel A			Panel B	
Variables	Observations	Mean	Std.	VIF	1/VIF
ROA	2,502	0.00912	1.01		
Current ratio	2,502	0.0197	1.046	1.25	0.797
Size	2,502	9.703	0.586	1.14	0.875
DR (capital structure)	2,502	0.5447	1.307	1.11	0.831
ROE	2,502	0.2859	0.766	1.21	0.824
Growth	2,502	0.271	0.167	1.20	0.831
HHI	2,502	0.8053	0.396	1.00	0.997
Innovation	2,502	0.0063	0.078	1.00	0.998
Mean VIF	1.13				

Panel B of Table 1 presents the VIF. Multicollinearity of the coefficients may lead to higher standard errors and makes the inference difficult and biased (Mamirkulova et al., 2020; Paulson et al., 2021; Zhou et al., 2021; Li et al., 2022). Therefore, to trace down the multicollinearity in this study, VIF confirms the absence of multicollinearity (Aman et al., 2019a,b, 2021a). Average values of all dependent and independent variables are lower than 10, confirming that our data are free from multicollinearity (Abbasi et al., 2021; Azadi et al., 2021; Local Burden of Disease HIV Collaborators, 2021; Wang et al., 2021). Previous studies stated that the value of VIF higher than five might indicate that a specific variable suffers multicollinearity (Hair et al., 2006; Li Y. et al., 2018). Panel B of Table 1 describes the details of the VIF analysis outlined below.

The article "Examining the Relationship Between Product Market Competition and Chinese Firms Performance: The Mediating Impact of Capital Structure and Moderating Influence of Firm Size" was retracted in 2025. Reasons: unreliable results or conclusions; a conflict of interest; concerns about the peer review; concerns about the citations.

### Analysis of Hypotheses 1 and 2

Hypothesis 1 showed that market competition and firm performance have a positive relationship. Thus, Table 2 reports the coefficient values of product market competition and firm performance. Model 1 displays that the coefficient values of HHI are0.619 and 0.300, respectively, with a 1% significant level with both performance measurements ROA and ROE. These results supported H1 of this study; there is a substantial and positive connection between product market competition and firm performance. Additionally, our outcomes are consistent with previous studies (Pant and Pattanayak, 2010; Ammann et al., 2013; Li M. et al., 2018).

**TABLE 2:** Market competition and firm performance: a mediating effect of capital structure.

Dependent variables	Model 1		Model 2	Model 3	
	ROE	ROA		ROE	ROA
HHI	0.619** (0.347)	0.30024** (0.150)		0.0858** (0.0446)	1.703*** (0.492)
D.R.			–0.0224*** (0.0076)	–0.0613*** (0.016)	–0.797*** (0.016)
R&D	–45.9* (35.03)	–0.270 (0.233)	20.78* (13.55)***	–15.14* (11.17)	–0.2843** (0.167)
Current ratio	3.368*** (0.685)	5.595*** (0.215)	–0.080** (0.041)	0.1310** (0.0683)	–0.549*** (0.104)
Growth	6.22 (1.608)	11.20*** (1.37)	–1.534** (0.649)	–0.7722*** (0.215)	–6.325*** (2.800)
Constant	–1.704*** (0.512)	–3.54 (0.337)	1.104*** (0.173)	0.5527*** (0.0783)	0.8085 (0.784)
Wald test	48.53***	24.25***	61.62***	45.38***	4,135***
AR (1)	–1.07	–1.02	–3.76	–3.78	–4.22
AR (2)	–1.75	–1.44	1.01	–1.78	0.29
Sargan test	4.08	6.86	118.04	719.21	202.04
Observation	2,502	2,502	2,502	2,502	2,502

***p < 0.01, **p < 0.05, *p < 0.1 shows significance levels.

Hypothesis 2 showed the mediating impact of capital structure on the association of market competition and firm performance. Model 2 specifies the outcomes of Hypothesis 2, which discloses the relationship between product market competition and capital structure. Model 2 describes that the GMM regression coefficient value is –0.0224 with a 1% significant level. This result showed that there is a negative association between capital structure and market competition. These outcomes confirmed our hypothesis from the other studies (Fosu, 2013). Therefore, leveraged businesses might suffer a substantial competitive difficulty in product markets because of high debt costs (Fosu, 2013). Additionally, Model 3 presents the consequences of the association between market competition and firm performance with the mediating effects of capital structure. Model 3 indicates the interaction term of HHI with both performance measurements ROA and ROE, respectively. Model 3 shows that the value of the coefficients of HHI is 0.0858 and 1.703 at 1% of significant level. These results supported H2.

The article "Examining the Relationship Between Product Market Competition and Chinese Firms Performance: The Mediating Impact of Capital Structure and Moderating Influence of Firm Size" was retracted in 2025. Reasons: unreliable results or conclusions; a conflict of interest; concerns about the peer review; concerns about the citations.

### Analysis of Hypothesis 3

Table 3 displays the outcomes of Models 4 and 5, which describe the association between product market competition and firm performance with the moderating role of firm size (small and large firm). Model 4 specifies the interaction term of small firms (S*HHI), with both performance measures. It shows the significant and negative coefficient value of S*HHI is –0.0676 and –0.2204, respectively. This result showed a statistically significant and negative connection between the small firm, capital structure, and firm performance. These outcomes indicate that small firms negatively moderate the relationship between product market competition and firm performance. The study results are consistent with other (Porter and Kramer, 2006; Javeed et al., 2021) outcomes, which stated that small firms have a low growth rate and profitability.

**TABLE 3:** Market competition and firm performance: a moderating effect of firm size.

Dependent variables	Model 4		Model 5	
	ROE	ROA	ROE	ROA
HHI	–0.0676** (0.39)	–0.2204*** (0.088)	0.1507*** (0.0527)	0.0405*** (0.0147)
Size	–0.0392* (0.149)	0.1258** (0.63)	0.4073*** (0.081)	0.0546** (0.0250)
S*HHI	0.2097*** (0.0625)	–0.0476 (0.064)		
L*HHI			–0.17092*** (0.062)	0.0231* (0.0219)
R&D	–0.1375*** (0.0420)	66.71*** (9.69)	0.1323*** (0.056)	–12.49*** (1.334)
Current ratio	0.1525** (0.0843)	0.1878*** (0.0501)	–0.0240 (0.077)	0.0688*** (0.020)
Growth	–0.5488* (0.361)	1.065** (0.508)	–4.237*** (1.55)	–0.1451 (0.160)
Constant	0.7587 (1.43)	–1.642*** (0.667)	–2.55*** (0.678)	–0.4658** (0.243)
Wald test	84.60***	19.31***	85***	19.4***
AR (1)	–3.92	–1.10	–4.39	–1.47
AR (2)	–1.65	–0.95	–1.64	1.00
Sargan test	203.08	85.10	17.84	587.68
Observation	2,502	2,502	2,502	2,502

***p < 0.01, **p < 0.05, *p < 0.1 shows significance levels.

Additionally, small organizations have limited products, and their managers do not consider innovative products, leading to low profits. Model 5 indicates the coefficient value of L*HHI is 0.1507 and 0.0405, statistically significant at 1% level. The positive coefficient value of L*HHI showed the positive role of large firms on market competition and firm performance. Large firms have more innovative and differentiated products that lead to higher profits. The results of Model 4 and 5 provide support for the proposed H3. See Table 3 below.

The article "Examining the Relationship Between Product Market Competition and Chinese Firms Performance: The Mediating Impact of Capital Structure and Moderating Influence of Firm Size" was retracted in 2025. Reasons: unreliable results or conclusions; a conflict of interest; concerns about the peer review; concerns about the citations.

## Discussion

H1 confirms the positive link between product market competition and firm performance, and previous literature supports our results (Javeed et al., 2020). Additionally, participating more in market competition can improve the company’s financial performance by establishing an excellent organizational image (Porter and Van der Linde, 1995). Companies in developing economies aim to improve market reputation and are considered unique, thereby bringing higher profits. The competition of developing economies forces companies to create innovative products and gain a first-mover advantage to maximize profits. Another study stated that high competition puts pressure on managers and makes them enthusiastic about making the company profitable when performing tasks (Raith, 2003). Thus, managers have limited opportunities to use firm resources for personal use in a highly competitive marketplace.

H2 indicates that capital structure mediates the association between product market competition and firm performance. Capital structure positively mediates this relationship, and outcomes are consistent (Fosberg, 2004). Existing literature demonstrated that leverage permits firms to compete in highly competitive environments, increasing shareholders’ benefits and leading to higher profits. Therefore, the capital structure allows a firm to gain competitive advantages by adding more products to achieve strategic objectives and maximize profit (Desai et al., 2003). Additionally, existing literature demonstrates that competitive benefit uncovers opportunities for opposition predation in a concentrated product marketplace. Thus, it leads to an increase in firm growth and profits. Previous studies have found the same outcomes and support our study (Abor, 2007).

H3 reports that firm size moderates the association between product market competition and firm performance. Product market competition and firm performance have a positive association with large firms. Our results are consistent with other studies’ (Porter and Kramer, 2006) outcomes, stating that large firms participate in CSR (other stakeholders) activities and create entry barriers for small businesses. This delivers higher benefits for large organizations. Furthermore, large firms always compel top firm executives to form a differentiated strategy for profit maximization. However, product market competition and firm performance have a negative association with small firms. Our results are consistent with (Porter and Van der Linde, 1995), which highlighted that the growth of small businesses and new product developments are slow, leading to a decline in profitability. Small businesses have limited products with the same revenue margin. Additionally, small firms use poor quality raw materials for making products and do not show innovative behavior leading to lower profitability (Dechezleprêtre and Sato, 2017). Furthermore, Raith (2003) added that small organizations keep managers more relaxed, decreasing profitability.

The article "Examining the Relationship Between Product Market Competition and Chinese Firms Performance: The Mediating Impact of Capital Structure and Moderating Influence of Firm Size" was retracted in 2025. Reasons: unreliable results or conclusions; a conflict of interest; concerns about the peer review; concerns about the citations.

The main benefits of competitive firms are that they have developed “global immunity” to the crisis by working in a highly turbulent environment for a long time, allowing them to remain resilient during the crisis (Iorember and Jelilov, 2018; Dabwor et al., 2020; Iorember et al., 2020; Maqsood et al., 2021; Mubeen et al., 2021; Liu et al., 2022). Government organizations and business firms encountered competitive environment in energy consumption demands, innovative products, global trade, and economic growth (Iorember and Jelilov, 2018; Iorember et al., 2019, 2021; Usman et al., 2019, 2020). The pandemic has developed challenges to meet renewable energy usage, human capital and quality environment (Usman et al., 2019, 2020; Jelilov et al., 2020; Iorember et al., 2021). Globally, the pandemic has posed household income inequalities, unemployment, and monitory policy shocks (Philip and Iorember, 2017; Goshit et al., 2020; Goshit and Iorember, 2020).

Business firms have faced challenges to protect their employees’ as vaccines availability for everyone was not guaranteed (Akhtar et al., 2020; Su et al., 2020, 2021a,b; Islam et al., 2021b). Companies encountered various challenges in the pandemic crisis (Anser et al., 2020; Akhtar et al., 2021a,b; Islam et al., 2021a). Business firms’ have seen tough competition to survive in the crisis (Akhtar et al., 2019b, 2021b; Siddiqi et al., 2019, 2020). Tourism and travel firms faced turbulent business environment to maintain their business growth in the competitive product market competition (Akhtar et al., 2019a; Ali et al., 2020; Ashraf et al., 2020; Siddiqi and Akhtar, 2020). Additionally, the companies benefited from their preparedness during the COVID-19 pandemic to safeguard their employees’ health with protective measures (Mohammadi et al., 2021; Shoib et al., 2021; Soroush et al., 2021; Liu et al., 2022). This ensures the entire industry’s sustainability, while all the advantages come from “competitive activities.” Another advantage is that competitive organizations allow companies to meet modern customers and environmental requirements that arose before the COVID-19 crisis and intensified during this period (additional services and digital solutions) (Pouresmaeil et al., 2019; Fattahi et al., 2020; Ilinova et al., 2021; Lebni et al., 2021). Further, competitive advantages allowed us to determine that they belong to “core competencies” and could be considered the basis for further growth in fertilizer companies. The key conclusion is that the competitive advantage could ensure the supply chain’s resilience and contribute to further growth. However, during a crisis, it is necessary to create core competencies to ensure growth. Thus the impact of the COVID-19 pandemic crisis on competitive fertilizer businesses is not crucial compared to other industries. The main factors of such resilience were: first, competitive firms play an important role and have always been turbulent. Therefore, they have some “immunity” to disturbances. Second, competitive organizations are strong and mature (Xu et al., 2021). This leads to the situation when the strength of competitors provides resilience to the entire industry. Third, competitive companies aim to create value for customers, shareholders, and society. However, competitive businesses transform by developing innovative tools, solutions, and technologies for growth (Zhou et al., 2021; Ge et al., 2022; Rahmat et al., 2022).

The article "Examining the Relationship Between Product Market Competition and Chinese Firms Performance: The Mediating Impact of Capital Structure and Moderating Influence of Firm Size" was retracted in 2025. Reasons: unreliable results or conclusions; a conflict of interest; concerns about the peer review; concerns about the citations.

## Conclusion

Many scholars have explored the direct relationship between product market competition and firm performance. Some positive relationships were found (Ruiz-Porras and Lopez-Mateo, 2011; Van Reenen, 2011; Javeed et al., 2020), while others were negative or U shape (Januszewski et al., 2002; Bloom et al., 2010; Ko et al., 2016). Thus, the literature did not explain the negative, positive, or neutral relationship between product market competition and firm performance. Furthermore, existing research demanded that omitted mediators and moderators be examined for studying the real effects of product market competition on firm performance (Guney et al., 2011; Sheikh, 2018). Consequently, based on these logical and rational claims, this study fills the literature gap by adding two associated variables, capital structure, and firm size, to show why and how product market competition influences company performance. After employing the GMM model, we concluded that product market competition and firm performance positively correlate.

The outcomes of our study show that competitive firms make innovative products and have limited probabilities to use firm resources for private benefits in a competitive market. This study examines the mediating impact of capital structure and finds that the capital structure positively mediates the relationship between product market competition and firm performance. The debt structure of firms uncovers opportunities for firms. Thus, it leads to an increase in firm growth and profits. Moreover, we investigated the moderating impact of firm size and found that large firms positively impact the association between product market competition and firm performance. As large organizations are well-reputed, they compel top firm executives to form a differentiated strategy for profit maximization. Additionally, the study tested small firms’ effects on the connection between product market competition and firm performance. This study found that small firms negatively affect the association of product market competition and firm performance. Moreover, it is stated that small firms do not show innovative behavior, leading to lower profitability (Dechezleprêtre and Sato, 2017).

The article "Examining the Relationship Between Product Market Competition and Chinese Firms Performance: The Mediating Impact of Capital Structure and Moderating Influence of Firm Size" was retracted in 2025. Reasons: unreliable results or conclusions; a conflict of interest; concerns about the peer review; concerns about the citations.

Based on this research, we provided suggestions for companies, decision-makers, and developed and developing economies to improve company performance. Our results will help the company attract owners, stakeholders, and investors to contribute to the competitive environment. The role of market competition and debt structure will be the focus of companies to increase profits. Our findings are helpful to decision-makers in formulating strategies in the industrial sector related to creating a competitive environment.

This study has several limitations. First, answer to the question how firm size moderates the product market competition and firm performance relationship is still unclear, which needs further theoretical development and thus helps us understand the mechanism of the moderating role in the relationship. Second, it is based on a sample of Chinese companies. A significant limitation may be China’s unique institutional environment. China is the second-largest economy globally due to its unique capital market and state intervention in the corporate sector. Therefore, the results of this study may not be generalized to other economies. However, few studies have been conducted from multiple aspects. On the contrary, these limitations provide the potential for future research and may help understand the link between competitive pressures and company performance. Future research could investigate the role of governance structure, corporate model, corporate governance, and finance allocation by selecting more data and sectors to understand the relationship between product market competition and company performance.

## Data Availability Statement

The original contributions presented in the study are included in the article/supplementary material, further inquiries can be directed to the corresponding authors.

## Author Contributions

RM and JA conceptualized the idea, contributed to study design, completed the entire article, including introduction, literature, discussion, conclusion, and edited the original manuscript before submission. DH reviewed and approved the final edited version and approved the submitted version. SR and WB have significantly helped and provided major contributions in revising this manuscript. They have also provided contribution to resource to make possible this manuscript. All authors reviewed and approved the final edited version and approved the submitted version.

The article "Examining the Relationship Between Product Market Competition and Chinese Firms Performance: The Mediating Impact of Capital Structure and Moderating Influence of Firm Size" was retracted in 2025. Reasons: unreliable results or conclusions; a conflict of interest; concerns about the peer review; concerns about the citations.

## Conflict of Interest

The authors declare that the research was conducted in the absence of any commercial or financial relationships that could be construed as a potential conflict of interest.

## Publisher’s Note

All claims expressed in this article are solely those of the authors and do not necessarily represent those of their affiliated organizations, or those of the publisher, the editors and the reviewers. Any product that may be evaluated in this article, or claim that may be made by its manufacturer, is not guaranteed or endorsed by the publisher.
